# The Expression of miR-205 in Prostate Carcinoma and the Relationship with Prognosis in Patients

This article has been retracted.

**DOI:** 10.1155/2022/1784791

**Published:** 2022-08-30

**Authors:** Zhuifeng Guo, Xuwei Lu, Fan Yang, Liang Qin, Ning Yang, Peiran Cai, Conghui Han, Jiawen Wu, Hang Wang

**Affiliations:** ^1^Department of Urology, Minhang Hospital, Fudan University, Shanghai, China; ^2^Center for Traditional Chinese Medicine and Gut Microbiota, Minhang Hospital, Fudan University, Shanghai, China; ^3^Department of Urology, Xuzhou Central Hospital, Xuzhou, Jiangsu, China; ^4^Department of Urology, Zhongshan Hospital, Fudan University, Shanghai, China

## Abstract

**Purpose:**

We aimed to investigate the changes of serum and cell exosome miR-205 levels in patients with prostate carcinoma and its clinical significance.

**Materials and Methods:**

Firstly, pronouncement of miR-205 in normal and prostate carcinoma tissues was analyzed by using UALCAN database. The relationship between miR-205 in tumor tissues and the pathological and clinical characteristics of patients with prostate carcinoma were analyzed. Consequently, 60 people with prostate carcinoma were collected to the Minhang Hospital from August 2016 to August 2021. Serum of patients in the two groups was collected, and RNA in serum exosomes was extracted, and qRT-PCR was used to analyze the expression of miR-205 mediated by serum exosomes. Meanwhile, the relationship among the clinical as well as pathological aspects and bodement of patients with prostate carcinoma and the pronouncement level of miR-205 mediated by exosome was compared. Next, assays like wound healing and CKK-8 were used to investigate the effects of miR-205 in exosomes extracted from prostate carcinoma on the augmentation and metastasis of prostate carcinoma.

**Results:**

The results showed that the pronouncement level of miR-205 in tissues with prostate carcinoma was significantly lower than that in normal prostate tissues. In addition, the pronouncement level of miR-205 in fluid exosome of people with prostate carcinoma and exosomes derived from the lines of prostate carcinoma was considerably less than that in serum exosomes of healthy patients and that of normal cell lines of prostate. The pronouncement level of miR-205 in fluid exosomes of people with prostate carcinoma was negatively associated with cancer phase, uncontrolled cell division in lymph nodes, distant metastasis, and PSA level at initial diagnosis. Analysis (multivariate and univariate) showed that miR-205 pronouncement was a sovereign threat cause for prognosis of prostate cancer patients. Additionally, the pronouncement and metastasis of prostate carcinoma can be restricted by the overexpression of miR-205.

**Conclusion:**

The pronouncement of miR-205 in liquid derived exosomes is correlated with the prediction of people with prostate carcinoma and may be a new marker for identification and cure of prostate carcinoma.

## 1. Introduction

Prostate cancer is the second largest virulence in males around the world, and in the genital and urinary system among males, it is the most common spreading lump [1].

Many prostate cancer patients do not respond to therapy through androgen stripping, and as a result, they are affected by a disease in which metastatic castration is permanent.

Early diagnosis and treatment can reduce the mortality and cost of patients. Screening for prostate cancer is usually done through two methods: first is the clinical manifestation, and the second one is test of serum prostate-specific antigen.

PSA screening often misdiagnoses certain ailments like hyperplasia in part prostate and prostatitis as carcinoma of prostate and leads to unnecessary invasive biopsy and overtreatment [2, 3]. PSA levels are also commonly used to monitor the recurrence of the disease, but the standard interval of PSA after radical surgery has been controversial. Therefore, there is a dire need of a new method to improve the quality of diagnosis of prostate cancer and the monitoring quality of progression of cancer.

Exosomes are actually some membraned vesicles like substances having about 30-150 nm diameter. They are released outside the cell after the mixing of cell membranes with the intracellular polyvesicles. They are mostly present in saliva, breast milk, amniotic fluid, blood, and urine. He et al. demonstrated that circulating exosomes in patients with SLE could be associated with disease activity and might therefore serve as biomarkers of disease activity [4]. Zhang et al. found that circulating exosomes suppressed the induction of regulatory T cells via let-7i-mediated blockade of the IGF1R/TGFBR1 pathway in multiple sclerosis [5].

Through recent experiments, it is proved that exosomes can be a medium for intracellular communication, and the content from donor cells such as DNA, mRNA, and miRNA can be transmitted towards the receiving cells in the future to regulate or interfere with specific physiological and pathological processes [6, 7]. Among RNAs contained in exosomes, miRNA content is the most abundant, and the types of miRNA in exosomes are selectively enriched, and their content directly reflects the expression level of miRNA in donor cells [8]. miRNAs are those RNAs which are noncoding. They are composed of 18-25 subunits called as nucleotides that results in the control of gene pronouncement after transcription [9, 10]. Each miRNA can regulate hundreds of transcripts through base complementary pairing, and the same transcript can bind more than one miRNA. Therefore, miRNA has a wide regulatory spectrum [11, 12]. In this study, the pronouncement levels of serum and cell exosome miR-205 in prostate cancer patients were analyzed to explore miR-205 amount in the early diagnosis and bodement test of prostate carcinoma, aiming to provide reference for the diagnosis and treatment of clinical diseases.

## 2. Methods and Materials

### 2.1. Clinical Specimens

A total of 60 prostate cancer patients admitted to the Minhang Hospital from August 2016 to August 2021 were objects in the research, and 60 healthy people were selected as the control group. Our study was approved by the Institutional Review Board of the Minhang Hospital, and written informed consent was obtained from each participant.

Inclusion criteria are as follows: (1) a participant had not injected with any form of anticarcinoma therapy before surgery. (2) All patients were confirmed by histopathological diagnosis of prostate cancer. (3) All patients or their family members understand the purpose and requirements of this study, agree to participate in this study, and sign consent in a printed form, and this study has been approved by the ethics committee of the Minhang Hospital. Elimination measures are as follows: (1) missing visitors or patients with incomplete clinical data; (2) patients with other tumors; and (3) complicated with severe cardiac, hepatic and renal insufficiency, and acute or chronic active pulmonary infection. The demographic characteristics and clinicopathological data of prostate cancer patients were recorded and summarized in Table 1.

### 2.2. Peripheral Blood Sample Collection

5mL of peripheral blood samples from tumor patients was extracted by anticoagulant tube, and the sample was extracted and kept at -80°C for subsequent experiments. Extract exosomes according to the instructions of the Exosome Extraction Kit (System Biosciences, USA) and do as follows: 500 *μ*L of serum sample was absorbed with a pipetting gun, and 126 *μ*L of extraction reagent was added and mixed by shaking. The serum was placed and incubated at 4°C for 30 min. The supernatant was removed by centrifugation, and 200 *μ*L of PBS was added for resuspension to obtain exosome suspension.

### 2.3. Extraction and Identification of Serum Exosomes

Cleared media were centrifuged at 100,000*g* for 70 min at 4°C following a method described previously [1]. The subsequent pellet was resuspended in PBS and washed three times by centrifugation at 100,000*g* for 70 min at 4°C. The clean pellet was then resuspended in 100 *μ*L of PBS or in NuPAGE™ LDS sample buffer. After polymerization at 60°C overnight, the precipitate was sliced, and the ultrathin sections were observed under a transmission electron microscope.

### 2.4. Extraction of RNA from Serum Exosomes

Follow the instructions for RNA extraction from serum exosomes (Qiagen, Valencia, CA, USA) kit. NanoDrop 2000 was used to detect RNA concentration, and a260/230 and A260/280 values and concentrations were recorded. If a260/230 value >2.1 (RNA degradation) and A260/280 <1.8, organic matter contaminated the extracted products.

### 2.5. The Extent of Pronouncement of miR-205 Mediated by Serum Exosome Was Detected by qRT-PCR

In accordance with the kit of TaqMan microRNA reverse transcription, there was a backward transcription of RNA into cDNA. The reaction conditions were as follows: reaction time was 15 min at 37°C, reaction 5 s at 85°C, and 4°C for 60 min. TaqMan microRNA Assay Kits (Applied Biosystems) are utilized to evaluate the pronouncement level of miR-205 in sample, which is mediated by exosome. PCR primers are miR-205: forward 5′-CTTGTCCTTCATTCCACCGGA-3′ and reverse 5′-TGCCGCCTGAACTTCACTCC-3′ and GAPDH: forward 5′-GAACGGGAAGCTCACTGG-3′ and reverse 5′-GCCTGCTTCACCACCTTCT-3′.

### 2.6. Cell Line Culture

Cell lines of patient with prostate tumor (DU145, 22RV1, and PC3) and RWPE-1 (normal prostatic epithelial cells) were acquired from Shanghai Yaji Biotechnology Co., Ltd. (Shanghai, China). RPMI-1640 medium or DMEM was used to incubate all the cells, and 10% FBS was the temperature for process of seeding at 37°C; they were cultured with 5% CO_2_.

### 2.7. Cell Transfection

PC3 cells at logarithmic growth stage were obtained, and trypsin was used for their digestion for 2-3 min. DMEM medium was used to make the suspension of cells and inoculated in 6-well culture plates for 6 h. Follow-up experiments were conducted when the cell density reached 50-80%. According to the Lipofectamine 2000 liposome kit specification, microRNA blank sequence (miR-205 NC) and miR-205 mimics (Shanghai Jima Biotechnology Co., LTD.) were transferred into prostate cancer PC3 cells, respectively. After routine overnight culture in the incubator, a mixture containing miR-205 mimics and transfection reagent was configured with a transfection concentration of 50 nmol/L. After reaction at room temperature for 30 min, the mixed reagents were added into 6-well culture plates, respectively, according to the grouping. After 4 h culture in the incubator at 37°C, the reagents were replaced with complete medium. Human prostate cancer cell line PC3 was collected from each group 24 h after transfection, and the extent of pronouncement of miR-205 was evaluated by qRT-PCR to detect the cell transfection efficiency. The RNA sequences were as follows: miR-205 NC: UUUGUACUACACAAAAGUACUG and miR-205 mimics: UCCUUCAUUCCACCGGAGUCUG.

### 2.8. Isolation of Cell Line Exosomes

Exosomes were extracted and purified from supernatant of cell culture collected super centrifugation from cell lines of prostate carcinoma and epithelial cell lines of normal prostate. The product was centrifuged at 300*g* for 10 min, at 2000*g* for 10 min, and at 10000*g* for 30 min. After each centrifugation, the supernatant was collected for the next centrifugation operation. The product was finally put in the centrifuge at 100000*g* for 70 min, and the product was wasted to collect sediment. After centrifugation at 100000*g* for 70 min, the precipitate was taken to obtain exosomes. Resuspended exosomes with 100 *μ*L PBS buffer should be stored in 4°C refrigerator when immediately used and stored in -80°C urtra-low temperature refrigerator when long-term storage. The ELISA kit is used for overall exosome capture and quantification (Biovision, ExoQuant™, Catalog # K1201).

### 2.9. Detection of Cell Proliferation Ability (CCK-8 Assay)

24 h after transfection, prostate cancer cells PC3 were digested with trypsin for 2-3 min and then inoculated into 96-well plates. 100 *μ*L was added to each well, with about 3 × 10^3^ cells. After incubating at 37°C for 0 h, 24 h, 48 h, 72 h, and 96 h, add CCK-8 solution 20 *μ*L/well to 6-well cells at each time and incubate at 37°C for 6 h, wavelength of enzyme plate was set at 450 nm of the microplate reader, absorbance of 96-well plate was measured, and growth curve was drawn. Repeat the experiment 3 times.

### 2.10. Detection of Cell Migration Ability (Wound Healing Assay)

First, use marker pen behind 6-hole plate, compare with ruler, equally make lines on the *x*-axis, with a continuous difference of 0.5-1 cm, across the hole, and the difference of each hole at least 5 lines. About 1 × 10^5^ cells were added into each well, and the specific number varied with different cell types. The inoculation principle was that the cell fusion rate reached 100% overnight. The next day with 200 *μ*L spear head than ruler, try to hang as far as the back of the horizontal line scratches; if the spear head is vertical, do not tilt. PBS was used for three times to clean the cells, the cells were removed, and medium without serum was added. After incubation at 37°C and 5%CO_2_ for 24 h, samples were taken and photos were taken. Finally, the migration distance of the two groups was compared.

### 2.11. Analysis Based on Statistics

The data was evaluated by utilizing SPSS 25.0, and for evaluation and mapping, we used GraphPad Prism 7.0 software. All measurement data in the form of mean ± standard deviation (SD), according to two groups and multiple groups of measuring data comparison using Student's *t*-test and analysis of variance (one-way). The relationship between the pronouncement of exosome miR-205 secreted by serum of people with prostate carcinoma and pathological and clinical manifestations of prostate carcinoma was examined through Pearson's chi-squared test, and the relationship amid the expression of miR-205 and the embodiment of prostate cancer patients was evaluated by the Kaplan-Meier survival analysis and Cox proportional hazard model. For a significant difference, *P* < 0.05 was selected.

## 3. Results

### 3.1. The Expression of miR-205 Was Significant Lower in the Prostate Tumor Tissues

Firstly, we used UALCAN database to analyze the pronouncement of miR-205 in prostate tumor tissues and normal tissues and revealed that the extent of pronouncement of miR-205 in c was significantly lesser than in normal prostate tissues (Figure 1(a)). Furthermore, the UALCAN database was used to evaluate the relationship between the pronouncement of miR-205 in prostate carcinoma tissues and the clinicopathological features of prostate cancer patients, and it was revealed that the relationship between miR-205 expression level in prostate cancer tissues and age, lymph node metastasis, and Gleason score was not statistically significant (Figures 1(b)–1(d)).

### 3.2. The Expression Level of Serum Exosome-Mediated miR-205 Is Negatively Correlated with Pathological as well as Clinical Features

The 120 serum samples (including 60 prostate cancer patient serum and 60 healthy subject serum) were selected to analyze the pronouncement of miR-205 in serum exosomes of people with prostate carcinoma by qRT-PCR. The findings suggested that the miR-205 pronouncement in serum exosomes of people with prostate tumor was lesser than that in serum exosomes of healthy patients (Figure 2(a)). To reveal the relationship between miR-205 expression and pathological and clinical manifestations of prostate carcinoma, the mentioned sections were divided into high (above the mean, *n* = 35) and low (below the mean, *n* = 25) miR-205 pronouncement classes (Figure 2(b)). The association between miR-205 pronouncement level and pathological and clinical manifestations of people with prostate tumor was analyzed using chi-squared test, and the findings revealed that the miR-205 pronouncement in serum exosomes of prostate tumor patients was significantly negatively linked with carcinoma stage, uncontrolled cell division in lymph node, distant metastasis, and PSA level at initial diagnosis in prostate cancer patients (Figures 2(c) and 2(d)), while the relationship with age of patients was not statistically significant (Table 1).

### 3.3. The Expression of miR-205 Pronouncement in Serum Exosomes Predicts Good Prognosis of Prostate Carcinoma

We firstly utilized the Kaplan-Meier survival analysis to investigate the correlation among miR-205 pronouncement in exosomes present in the serum of people with prostate cancer and prognosis of patients with prostate cancer. The findings revealed that the inclusive survival rate of people with more miR-205 pronouncement in serum exosomes was higher than that of people with less miR-205 pronouncement (Figure 3), which suggested that miR-205 in serum exosomes played a significant part in the prognosis of patients with prostate tumor. Next, we conducted COX proportional risk model analysis, and the findings of univariate analysis showed that carcinoma stage, PSA level at initial diagnosis, and miR-205 pronouncement were significantly correlated with the inclusive survival rate of people with prostate carcinoma. Furthermore, the results of multivariate investigation indicated that miR-205 utterance in serum exosomes was an impartial risk aspect for prognosis in people with prostate tumor (Table 2).

### 3.4. The miR-205 Extent of Pronouncement in Exosomes Extracted from Prostate Carcinoma Cell Lines

Cell lines of prostate tumor (DU145, 22RV1, and PC3) and normal prostatic cell line of epithelium RWPE-1 were selected to analyze the miR-205 expression in exosomes derived from cell lies of prostate carcinoma by qRT-PCR. The findings suggested that the miR-205 pronouncement in exosomes of prostate cancer cell lines was significantly lower than that in exosomes of normal cell line of epithelium (Figure 4(a)).

### 3.5. The miR-205 Promotes the Spread and Migration of Prostate Carcinoma Cells

In order to further study the role of miR-205 in prostate carcinoma cells, in this study, the miR-NC and miR-205 mimics were transfected into PC3 cell line, and the RT-PCR was applied to identify cell transfection efficiency of miR-205. The findings revealed that contrasted with miR-NC group, after transfection with miR-205 mimics, the pronouncement level of miR-205 in PC3 was higher with statistically significant difference (Figure 4(b)). Subsequently, proliferation and migration experiments were conducted, and the results of proliferation detection revealed that overexpression of miR-205 could significantly activate the spread of prostate carcinoma linked with the miR-NC class (Figure 4(c)). In addition, the migration detection findings revealed that overexpression of miR-205 promoted the migration of prostate cancer cells contrasted with the miR-NC group (Figure 4(d)).

## 4. Discussion

Prostate cancer is one of the extremely widespread cancerous growths in the genitourinary system in elderly men. Its death rate and morbidity rate rank the 2nd and 5th in the global malignant tumor incidence and mortality spectrum, the 1st and 3rd in men in Europe and America, and the 6th and 7th in men in China, respectively [1, 13]. In recent years, with the aging of China's population and other reasons, the incidence and death of prostate cancer have increased significantly, and the disease burden is increasing [14, 15]. Prostate-specific antigen is commonly used biomarker for the screening of prostate carcinoma, but it cannot distinguish the benign and malignant prostate diseases well [16–18]. The Gleason histopathological score is used to assess the prognosis of patients, who often experience additional pain due to invasive procedures [19, 20]. Therefore, highly specific and noninvasive biomarkers are required to lead the analysis and cure of prostate cancer on urgent basis.

Exosomes are vesicles present outside the cell. They have a diameter of 30-150 nm and lipid bilayer membrane, which are mostly found in numerous body liquids [21, 22]. The main substances of exosomes include proteins, nucleic acids, and lipids. Exosomes secreted by different tissues have different compositions [23]. The lipid bilayer structure of exosomes can protect its contents from degradation by protease and RNA enzyme, and it has high biological stability. Protein is the main component of exosome content, which can directly change the invasion and relocation capability of tumor carcinoma and stimulate tumor progression and uncontrolled cell division [24]. Nucleic acids in exosomes, including mRNA, miRNA, and DNA, can be transferred and change the receptor cell signaling pathway through the fusion of exosomes and target cell membranes [25, 26].

Recent studies have found that miRNAs carried by exosomes derived from cancer cells are engaged in the genesis, angiogenesis, invasion, and uncontrolled cell division of nasopharyngeal carcinoma, breast carcinoma, and other tumor tissues [27, 28]. Prostate cancer cells create a microenvironment conducive to tumor growth by releasing exosomes containing specific components. The miR-424 in exosomes secreted by prostate cancer could induce tumor transformation of normal prostate epithelial cells and further promote the progression of the disease through intercellular transmission, and miR-183 in exosomes secreted by prostate cancer could indorse the propagation, invasion, and uncontrolled cell divisions of cancer cells by downregulating TPM1 pronouncement [29, 30].

Human miR-205 is in the LOC642587 gene of chromosomal lq32.2, which has significant tissue specificity and can be particularly shown in human thymus, breast, prostate, and other tissues, and can control the appearance of multiple target genes. It is involved in the proliferation, apoptosis, differentiation, angiogenesis, drug resistance, infiltration, and uncontrolled cell division of tumor cells. Moreover, miR-205 is expressed differently in different cancer tissues, with high expression in bladder cancer, ovarian cancer, and lung cancer, but low expression in breast cancer, and no difference in colon cancer tissue, indicating that miR-205 cannot only indorse the incidence and growth of lump as a carcinogen miRNAs. It can also be involved in the occurrence and development of tumors as tumor suppressor miRNAs [31, 32]. To study the link between miR-205 pronouncement level and prognosis in prostate cancer, we first examined the UALCAN database and discovered that the pronouncement level of miR-205 in prostate carcinoma tissues was lesser than that in normal prostate tissues. Next, we selected 120 serum samples to analyze the miR-205 pronouncement in serum exosomes of people with prostate carcinoma, and the results suggested that the miR-205 pronouncement in serum exosomes of people with prostate carcinoma was significantly lesser than that in serum exosomes of healthy people. Furthermore, the miR-205 utterance in serum exosomes of people with prostate carcinoma was significantly negatively connected with tumor stage, uncontrolled cell division in lymph node, distant metastasis, and PSA level at initial diagnosis in prostate cancer patients and could be used as a sovereign risk aspect for prognosis in people with prostate carcinoma. In addition, we also found that the miR-205 expression in exosomes of prostate carcinoma cell lines was significantly less than that in exosomes of normal human prostatic cell line of epithelium, and miR-205 could encourage the proliferation and migration of prostate tumor cells. Our results suggested that miR-205 could be implicated in the incidence and progress of prostate tumor as tumor suppressor miRNAs.

## 5. Conclusion

The pronouncement of miR-205 mediated by serum exosomes and cell exosomes in prostate cancer patients can be used as an indicator of tumor progression and poor prognosis and also indicates that exosome-mediated miRNA may be utilized as biological markers for early analysis and prediction of malicious carcinomas.

## Figures and Tables

**Figure 1:** The miR-205 expression in the database. (a) The miR-205 expression in prostate tumor tissues and normal tissues. (b) The relationship between the expression of miR-205 expression and age in prostate cancer tissues. (c) The relationship between miR-205 expression and lymph node metastasis in prostate cancer tissues. (d) The relationship between miR-205 expression and Gleason score in prostate cancer tissues.

**Figure 2:** The miR-205 expression in exosomes extracted from prostate carcinoma cell lines and the biological function. (a) The miR-205 expression in exosomes extracted from prostate carcinoma cell lines and normal prostatic cell line of epithelium. (b) The miR-205 expression in exosomes extracted from miR-NC group and miR-205 mimics. (c) The miR-205 promotes the proliferation of prostate cancer cells. (d) The miR-205 promotes the migration of prostate cancer cells. ^∗^*P* < 0.05, ^∗∗^*P* < 0.01, and ^∗∗∗^*P* < 0.001 (Student's *t*-test). Abbreviations: HR: hazard ratio; CI: confidence interval.

**Figure 3:** The relationship between the expression level of serum exosome-mediated miR-205 and pathological, clinical features in prostate cancer patients. (a) The miR-205 expression in serum exosomes of people with prostate tumor and healthy patients. (b) The miR-205 expression was divided into high (above the mean, *n* = 35) and low (below the mean, *n* = 25) miR-205 expression classes. (c) The relationship between the expression level of serum exosome-mediated miR-205 and carcinoma stage, lymph node metastasis in prostate carcinoma. (d) The relationship between the expression level of serum exosome-mediated miR-205 and distant metastasis, PSA level in prostate carcinoma at initial diagnosis. ∗*P* < 0.05, ^∗∗^*P* < 0.01, and ^∗∗∗^*P* < 0.001 (Student's *t*-test).

**Figure 4:** The relationship between miR-205 expression in serum exosomes of people with prostate cancer and prognosis of patients.

**Table 1:** The relationship between the expression of exosome miR-205 secreted by serum of prostate cancer patients and clinicopathological features of prostate cancer patients (*n* = 60).

Characteristics	miR-205 expression		Chi-squared test	*P* value
	Low no. cases	High no. cases		
All patients	(*n* = 25)	(*n* = 35)		
Age(years)			0.156	0.693
≤60	13	20		
>60	12	15		
Tumor stage			9.16	0.002
≤T2	8	25		
>T2	17	10		
Lymph node metastasis			5.173	0.023
Negative	9	23		
Positive	16	12		
Distant metastasis			7.837	0.005
M0	8	24		
M1	17	11		
PSA at initial diagnosis (ng/mL)			11.051	0.001
≤20	7	25		
>20	18	10		

**Table 2:** Univariate and multivariate analysis of overall survival in patients with prostate cancer (*n* = 60).

Variable for overall survival	Univariate analysis			Multivariate analysis		
	HR	95% CI	*P*	HR	95% CI	*P*
Age(years)			0.897			
≤60 vs. >60	1.043	0.547-1.989				
Lymph node metastasis			0.071			
Negative vs. positive	1.819	0.950-3.485				
Distant metastasis			0.218			
M0 vs. M1	1.501	0.786-2.863				
Tumor stage			0.011			0.105
≤T2 vs. >T2	2.364	1.220-4.580		0.565	0.283-1.128	
PSA at initial diagnosis (ng/mL)			0.008			0.294
≤20 vs. >20	2.45	1.263-4.754		0.671	0.318-1.414	
miR-205 expression			*P* < 0.001			0.021
Low vs. high	3.251	1.675-6.313		0.417	0.198-0.878	

## Data Availability

The data could be obtained from contacting the corresponding author.
